The article "Clinical Study on the Relationship between the SNP rs8192675 (C/C) Site of SLC2A2 Gene and the Hypoglycemic Effect of Metformin in Type 2 Diabetes" was retracted in 2022. Reason: concerns about the peer review.

# Clinical Study on the Relationship between the SNP rs8192675 (C/C) Site of SLC2A2 Gene and the Hypoglycemic Effect of Metformin in Type 2 Diabetes

**DOI:** 10.1155/2022/3645336

**Published:** 2022-01-31

**Authors:** Weiwei Ye, Yi Wang, Feng Chen, Qian Zhao, Xiangying Meng, Jianyang Chen, Cong Liu, Yong Zhou

**Affiliations:** Department of Endocrinology, Dahua Hospital, Xuhui, Shanghai 200237, China

## Abstract

This study investigates the correlation between the gene polymorphism of rs8192675 (C/C) locus of SLC2A2 in patients with type 2 diabetes (T2DM) and the efficacy of metformin. For this purpose, we have selected 110 T2DM patients (T2DM group) and 110 healthy people (control group) who were treated in our hospital from January 2019 to January 2020 as the research subjects. PCR-restriction fragment length polymorphism (PCR-RFLP) method detects the distribution frequency of gene polymorphism. The patients in the T2DM group were treated with metformin and followed up for 90 days to analyze the relationship between the efficacy of metformin and the SLC2A2 gene polymorphism. The genotypes of SLC2A2 rs8192675 in the control group and in the T2DM group conformed to the Hardy–Weinberg equilibrium law. Compared with the control group, the CT type and the CC type at rs8192675 in the T2DM group were significantly higher (*P* < 0.05). For rs8192675, there was no significant difference in TT, CT, CC FPG, 2hPBG, and HbA1c levels before treatment (*P* > 0.05); after metformin treatment, the reduction in FPG, 2hPBG, and HbA1c in CC patients was lower than that of TT and CT patients (*P* < 0.05). SLC2A2 gene polymorphism site rs8192675 CC type T2DM patients are sensitive to metformin and have a better hypoglycemic effect.

## 1. Introduction

Diabetes mellitus is a group of metabolic diseases characterized by increased chronic blood sugar levels, which are caused by defects in insulin secretion and/or function. Due to long-term carbohydrate, fat, and protein metabolism disorders, multiple systems of the body are damaged, which can eventually lead to chronic progressive disease, hypofunction, and failure of various tissues and organs, which seriously affect the quality of life of patients, reduce the life span of patients, and increase the mortality rate of patients. Among the rapidly growing diabetic patients, type 2 diabetes mellitus (T2DM) patients account for the vast majority. At present, it is believed that insulin resistance and insulin secretion defects are the basis of their onset, which can occur at any age, more often than 35-year-old adult. Its pathogenesis is mainly manifested in insulin resistance and *β*-cell function defects, and insulin resistance appears earlier in the pathogenesis. T2DM is caused by a combination of multiple factors, including genetic and environmental factors. In 2005, O'Rahilly S published an article in science that pointed out that genetic factors occupy a major position [1]. Insulin gene , KCNJ11, TCF7L2, SLC30A8 proliferator receptor gene [2–6], etc., are all related to the polymorphism of T2DM-related genes.

Oral hypoglycemic agents such as alpha-glycosidase inhibitors and insulin sensitizers are commonly used in the clinical treatment for T2DM; metformin was approved by the US FDA in 1994 and recommended as the first-line treatment for T2DM by most guidelines, becoming a secondary sulfonylurea, the most widely used oral hypoglycemic agent after the class of drugs. Its hypoglycemic mechanism is to increase the sensitivity of surrounding tissues to insulin, inhibit hepatic gluconeogenesis, and at the same time inhibit the uptake of glucose by intestinal wall cells. Overweight patients with T2DM are often the first choice for the treatment with metformin, which can prevent vascular complications and reduce mortality while controlling blood sugar. The effect is better than other oral hypoglycemic drugs and diet control [7]. Studies have shown that adenosine phosphate-activated protein kinase (AMPK) is the main cell regulator of lipid and glucose metabolism. Metformin acts by activating AMPK [8], and this effect may be related to the AMPK signal transduction system. In the body, metformin can inhibit the mitochondrial respiratory chain, thereby changing the ratio of ATP to AMP in the cell, indirectly activate AMPK, inhibit liver gluconeogenesis, have a negative impact on lipid synthesis, and promote the uptake and utilization of glucose by skeletal muscle [9, 10].

Human disease-causing gene polymorphisms play an important role in response to drug treatments; that is, disease gene polymorphisms can affect the drug metabolism process, so that patients with different genotypes have different responses to drugs [11]. Proximal tubular glucose transporter 2 (SLC2A2) is a high-efficiency glucose transporter, expressed in liver, kidney, intestine, and pancreatic cells. Studies have shown that the relationship between SLC2A2 gene polymorphism and metformin treatment of T2DM patients is less.

This study investigates the correlation between the gene polymorphism of rs8192675 (C/C) locus of SLC2A2 in patients with type 2 diabetes (T2DM) and the efficacy of metformin. For this purpose, we have selected 110 T2DM patients (T2DM group) and 110 healthy people (control group) who were treated in our hospital from January 2019 to January 2020 as the research subjects. PCR-restriction fragment length polymorphism (PCR-RFLP) method detects the distribution frequency of gene polymorphism. The patients in the T2DM group were treated with metformin and followed up for 90 days to analyze the relationship between the efficacy of metformin and the SLC2A2 gene polymorphism.

The remaining paper is organized as given below in the agenda items.

In the subsequent section, that is, Section 2, materials and methodology, which are used to realize the proposed scheme, are described and depicted in detail. In Section 3, various observations and achievements of the proposed system, which are verified through extensive experiments, are presented in both textual and graphical formats. Finally, concluding remarks are provided in the last section along with possible future directions.

## 2. Materials and Methods

### 2.1. Main Reagents

The main reagents used are as follows: physiological saline (Hubei Xinghua Pharmaceutical Co., Ltd.); sterilized plasma water (laboratory self-made); DNA extraction solution of 10% NH4CL (Beijing China Times Gene Technology Development Co., Ltd.); DNA preservation solution (Yao Jinbao: Beijing China Times Gene Technology Development Co., Ltd.); sequencing reaction universal kit (Yaojin points: Beijing China Times Gene Technology Development Co., Ltd.); glucose determination kit (Anhui Daqian Bioengineering Co., Ltd.); insulin determination kit (Siemens, USA); and glycosylated hemoglobin A1c detection kit (Bio-Rad Laboratories, Inc.).

### 2.2. Main Instruments

The main instruments used are as follows: vortex mixer (Jiangsu Kangjian Medical Products Co., Ltd., XH-D); high-speed centrifuge (Anhui Zhongke Zhongjia Scientific Instrument Co., Ltd., HC-2516); handheld centrifuge (Qilin Bell Instrument Manufacturing Co., Ltd., LX-400); real-time fluorescent quantitative PCR instrument (Xi'an Tianlong Technology Co., Ltd., RT-CyclerTM436/TL998 A); centrifuge (Anhui Zhongke Zhongjia Scientific Instrument Co., Ltd., KDC-1042); fully automated chemiluminescence immunoassay analysis system (Siemens, ADVIA Centaur XP, USA); automatic hemoglobin test system (Bio-Rad Laboratories, Inc., ARIANT II); and automatic hematology analyzer (Sysmex, XN 9000).

### 2.3. Proposed Methodology

#### 2.3.1. General Information

The test subjects were 110 patients with type 2 diabetes (T2DM) who were first diagnosed in our hospital from January 2019 to January 2020, including 50 males and 47 females; they were 20 to 75 years old, with an average age of 58.2 ± 14.0 years. All subjects were not related, and all subjects signed an informed consent form.

#### 2.3.2. Enrollment Criteria

1. If one of the following conditions is met arbitrarily and confirmed repeatedly, the diagnosis is established: newly diagnosed type 2 diabetes patients who meet the 1999 WHO Diabetes Diagnostic Standards, that is, diabetic symptoms (polydipsia, polyuria, polyphagia, decreased body weight), plus random blood glucose test ≥11.1 mmol; FPG (fasting blood glucose) ≥7.0 mmol/L; or blood glucose test ≥11.1 mmol 2 h after adding glucose load
2. The age is over 16 years
3. Fasting blood glucose is between 7.0 and 18.0 mmol/L
4. Height and body mass index (BMI) are 18.5–27.5 kg/m^2^
5. No history of oral hypoglycemic drugs or insulin therapy in the last 15 days

#### 2.3.3. Exclusion Criteria

1. Renal insufficiency (blood creatinine level> 132.6 *μ*mol/L (1.5 mg/dL) for men, > 123.8 *μ*mol/L (1.4 mg/dL) for women or estimated glomerular filtration rate (GFR) < 45 mL/min), liver insufficiency, severe infection, hypoxia or patients undergoing major surgery, diabetic hyperosmolar coma, ketoacidosis, and severe cardiovascular disease
2. Acute or chronic cardiac insufficiency people, and blood diseases
3. Pregnant and lactating women
4. Alcoholics

#### 2.3.4. Criteria for Discontinuation of the Experiment

1. If the patient has an increase in blood lactic acid> 3 mmol/L, urine ketone body, blood creatinine> 120 mmol/L, and the urine ketone is positive, the drug should be stopped immediately, and the clinical trial should be stopped according to the doctor's judgment
2. patients with angina pectoris, myocardial infarction, intermittent claudication, sepsis, and deterioration of heart, lung, liver, and kidney functions should all be discontinued
3. patients have poor compliance and missed medication for 10 days or more
4. subjects voluntarily asked the doctor to suspend during the clinical trial due to personal reasons

#### 2.3.5. Dosing Schedule

The patient took metformin hydrochloride tablets, and the course of study and observation was 90 days. Fasting blood glucose, fasting insulin, and glycated hemoglobin before and after treatment were monitored, and drinking alcohol is avoided. The dose of the drug is adjusted every 15 days: if the patient has FPG ≥7 mmol/L, 500 mg/d, or 750 mg/d, the dose will be doubled, 1000 mg/d will be increased to 1500 mg/d, and the maximum dose will be 2 500 mg/d; if FPG<7.0 mmol/L, this dose is continued and maintained until the end of follow-up. If adverse gastrointestinal reactions related to metformin occur during the medication and the medication does not improve after 4–10 days, the dose can be lowered or the medication may be stopped as appropriate.

#### 2.3.6. Detection of SLC2A2

Gene polymorphism: a 2 mL EDTA anticoagulant tube was used for the collection of subjects' venous blood. SLC2A2 genotype detection adopts the fluorescence in situ hybridization (FISH) method, one of the nine sequencing methods recommended in the National Health Commission's “Drug Metabolism Enzyme and Drug Target Gene Detection Technology Guide (Trial).”

### 2.4. Statistical Analysis

Statistical software SPSS Statistics 22.0 was used for statistical data analysis. The measurement data were expressed as mean ± standard deviation (*x* ± *s*), and the comparison between the two groups was performed by *t*-test; the count data were expressed by *n,* and the chi-square test was used; and the Hardy–Weinberg genetic balance test was used as a degree of balance. The data are all *P* < 0.05 representing statistical differences.

## 3. Experimental Results

### 3.1. Hardy–Weinberg Equilibrium Law

According to the Hardy–Weinberg equilibrium law, the expected value and observed value of each genotype of SLC2A2 rs8192675 locus in the control group and in the T2DM group were tested, and they were all *P* > 0.05, which conformed to the Hardy–Weinberg equilibrium law, suggesting that the population is from the same Mendelian population, selected. The sample is the representative of population genetic research, and the results are shown in Table 1.

### 3.2. SLC2A2 Gene Polymorphism Site rs8192675 Polymorphism Analysis

Compared with the control group, the CT type and the CC type at rs8192675 in the T2DM group were significantly higher (*P* < 0.05), as shown in Table 2.

### 3.3. Relationship between SLC2A2 and the Efficacy of Metformin in Patients with T2DM

For the rs8192675 locus, there was no significant difference in the levels of TT, CT, CC FPG, 2hPBG, and HbA1c before treatment (*P* > 0.05); after metformin treatment, the reduction in FPG, 2hPBG, and HbA1c in CC patients was lower than that of TT and CT patients (*P* < 0.05) (see Tables 3, 4, and 5 and Figure 1 for details).

The participants were stratified into the obese (BMI≥30 kg/m^2^) and nonobese (BMI<30 kg/m^2^) groups. The error bars are for the standard error of the mean HbA1c reduction.

## 4. Discussion

Diabetes is a group of metabolic diseases with hyperglycemia and insulin resistance, which tend to increase the incidence of serious diseases in various systems of patients. At the same time, this situation will also bring harm to the patient's quality of life and economic burden [12]. Prolonged hyperglycemia can cause serious damage to microvessels and further increase the incidence of various complications [13]. The International Diabetes Federation (IDF) reported that in 2017, the number of adults with type 2 diabetes reached more than 424.9 million, and the number of patients with type 2 diabetes is expected to increase to 629 million by 2045 [14]. Since the major guidelines proposed that the key drug for diabetes is metformin [15, 16], metformin has been considered the most commonly used oral hypoglycemic agent at present. However, it has been found in clinical practice that there are certain individual differences in its drug treatment, which may be mainly caused by genetic factors. Among them, transporter polymorphism has become the focus of current metformin genetic pharmacology research [17].

Metformin is widely used in clinical practice. Metformin can be used as a single agent to treat T2DM, or it can be combined with other oral hypoglycemic drugs or insulin. However, the molecular mechanism of lowering blood sugar is not very clear today. Research results have now shown that metformin acts on liver cells to reduce the glucose production in the liver, inhibit liver glycogen decomposition, and improve the insulin sensitivity of glucose metabolism in the muscles, thereby reducing blood sugar in patients with T2DM. Studies have shown that AMPK is the main cell regulator of lipid and glucose metabolism, and metformin works by inhibiting AMPK. After being taken orally into the body, metformin does not undergo liver metabolism and bile excretion, but is excreted in the form of prototype through urine. It is mainly excreted in the kidney in the form of tubular secretion, and the renal clearance rate is greater than the glomerular filtration rate. A variety of organic cation transporters are key factors in the transport and distribution of metformin in the body. For a long time, various studies have believed that drug-metabolizing enzymes and drug receptors affect the metabolic transport of drugs in the body. Nowadays, the important role of various membrane transporters in the metabolic transport of drugs has attracted more and more attention and reports.

The SLC2A2 gene is located at q26.1∼q16.2 on chromosome 3, and the encoded protein can regulate the transport factor of glucose into the cell. Studies have shown that mutations in the SLC2A2 gene can lead to abnormal protein function, leading to abnormal glucose metabolism in the body. SLC2A2 encodes the glucose transporter isoform GLUT2, which is expressed in liver, kidney, intestine, pancreatic *β* cells, and central nervous system (neurons, astrocytes) [18]. It is believed that the hypoglycemic effect of metformin mainly comes from reducing hepatic glucose output by inhibiting gluconeogenesis and also from increasing muscle glucose uptake [19]. In addition, metformin may also play a role by changing the gut microbiome [19]. Gene expression data from 1,226 human liver samples showed that people with the C allele had reduced SLC2A2 expression, which is likely to cause a decrease in GLUT2 activity in the liver [20]. This genetic change may be actively regulated by metformin. One possible explanation for this finding may be that C allele carriers have reduced glucose clearance, including a reduced ability for glucose to enter the liver, and metformin treatment can improve this situation. In addition, GLUT2 is also responsible for the release of liver glucose [21]. It is conceivable that people with the C allele variant of the SLC2A2 gene may be more sensitive to the effects of metformin on the liver. In early type 2 diabetes, insulin secretion usually increases due to the prevalence of insulin resistance [22]. Over time, insulin secretion will increase and begin to decrease, and blood sugar control deteriorates [22].

This study shows that the SNP rs8192675 in the SLC2A2 gene (C allele) was associated with an improved glucose response to metformin monotherapy in patients with newly diagnosed type 2 diabetes. These findings are in line with a three-stage genome-wide association study including 13,123 type 2 diabetes patients from the MetGen Consortium, which reported that having a C allele was related to higher baseline HbA1c values independent of the type of glucose-lowering therapy and to a significantly larger on-treatment HbA1c reduction for metformin users only [18]. SLC2A2 encodes the glucose transporter isoform GLUT2, which is expressed in liver, kidney, intestine, pancreatic islet beta cells, and the central nervous system (neurons, astrocytes) [20]. The glucose-lowering effect of metformin is believed to result mainly from decreased hepatic glucose output through inhibition of gluconeogenesis, but also from increased muscle glucose uptake [19]. Furthermore, metformin may also act through alterations in the gut microbiome [19]. Gene expression data from 1226 human liver samples revealed that SLC2A2 expression is decreased in people with the C allele, which most likely results in less GLUT2 activity in the liver. This genetic alteration may be positively modulated by metformin. A possible explanation for the present finding could be that glucose clearance is reduced in C allele carriers, including a decreased ability of glucose to enter the liver, which is improved by metformin therapy. Furthermore, GLUT2 is also responsible for hepatic glucose release [21]. It is conceivable that people with the C allele variant of the SLC2A2 gene may be more sensitive to the effects of metformin on the liver. In early type 2 diabetes, insulin secretion is commonly increased because of the prevailing insulin resistance [22]. Over time, insulin secretion begins to decline and glycaemic control worsens [22]. In this study, neither C-peptide stimulation nor glucose disappearance rate was increased in C allele carriers with metformin monotherapy. It is noteworthy that it has previously been reported that metformin improves glucose disappearance as assessed by IVGTT in women with polycystic ovary syndrome.

Our results should be interpreted in the context of some limitations. First, the data on diabetes-related symptoms and fasting glucose values at the time of diabetes diagnosis relied on self-reports only. Second, metformin blood concentrations were not measured. Third, while the primary endpoint was the change in blood glucose from diagnosis to baseline, for various other variables there were no data available at the time of diabetes diagnosis. Therefore, the corresponding tests and *p* values should be interpreted as hypothesis-generating [23].

## 5. Conclusion and Future Directions

In this study, we have investigated the correlation between the gene polymorphism of rs8192675 (C/C) locus of SLC2A2 in patients with type 2 diabetes (T2DM) and the efficacy of metformin. For this purpose, we have selected 110 T2DM patients (T2DM group) and 110 healthy people (control group) who were treated in our hospital from January 2019 to January 2020 as the research subjects. PCR-restriction fragment length polymorphism (PCR-RFLP) method detects the distribution frequency of gene polymorphism. The patients in the T2DM group were treated with metformin and followed up for 90 days to analyze the relationship between the efficacy of metformin and the SLC2A2 gene polymorphism. The results showed that the genotypes of SLC2A2 rs8192675 in the control group and in the T2DM group conformed to the Hardy–Weinberg equilibrium law. Compared with the control group, the CT type and the CC type at rs8192675 in the T2DM group were significantly higher (*P* < 0.05). For rs8192675, there was no significant difference in TT, CT, CC FPG, 2hPBG, and HbA1c levels before treatment (*P* > 0.05); after metformin treatment, the reduction in FPG, 2hPBG, and HbA1c in CC patients was lower than that in TT and CT patients (*P* < 0.05). The above studies have proved that the SLC2A2 gene polymorphism site rs8192675 CC type T2DM patients are sensitive to metformin and have a better hypoglycemic effect.

In future, we are eager to extend the proposed model to check the sensitivity of other patients or group of people from different perspectives.

## Figures and Tables

**Figure 1:** HbA1c reduction by the BMI group and rs8192675 genotype.

**Table 1:** Hardy–Weinberg genetic balance test results (N).

Genotype	Control group (*n* = 110)		X^2^	*P*	T2DM group (*n* = 110)		X^2^	*P*
	Observation value	Expected value			Observation value	Expected value		
TT	89	85.5	2.135	0.356	68	66.8	2.861	0.126
CT	15	18.6			30	35.9		
CC	6	5.9			12	7.3		

**Table 2:** Genotype distribution of SLC2A2 locus in the control group and in the T2M group (%).

Group	Number of cases	Genotype			Allele	
		TT	CT	CC	A	C
Control	110	89	15	6	193 (87.7)	27 (12.3)
T2DM	110	68	30	12	166 (75.5)	54 (24.5)
X^2^		15.602	8.890	7.890	21.361	
P		0.000	0.002	0.003	0.000	

**Table 3:** Relationship between SLC2A2 genotype and metformin efficacy (FBG value) in patients with T2DM (*X* ± *S*).

Genotype	Number of cases	FBG		t value	*P* value
		Before treatment	After treatment		
TT	68	10.21 ± 1.56	8.21 ± 1.29	1.236	0.000
CT	30	10.12 ± 1.58	7.16 ± 1.18^a^	3.256	0.006
CC	12	9.98 ± 1.55	6.29 ± 1.09^ab^	12.365	0.235
F value		0.029	20.365		
*P* value		0.869	0.000		

*Note.* FBG is fasting plasma glucose, 2hPBG is 2h postprandial blood glucose, HbA1c is hemoglobin A1c; compared with TT type, ^a^*P* < 0.05; compared with CT type, ^b^*P* < 0.05.

**Table 4:** Relationship between SLC2A2 genotype and the efficacy of metformin (2hpbc value) in T2DM patients (*X* ± *S*).

Genotype	Number of cases	HbA1c		t value	*P* value
		Before treatment	After treatment		
TT	68	15.22 ± 2.56	14.10 ± 2.25	1.236	0.239
CT	30	14.39 ± 2.51	13.71 ± 2.29^a^	2.038	0.046
CC	12	15.39 ± 2.48	12.39 ± 2.14^a^	5.689	0.000
F value		1.226	8.195		
*P* value		0.871	0.001		

*Note.* FPG is fasting plasma glucose, 2hPBG is 2h postprandial blood glucose, HbA1c is hemoglobin A1c; compared with TT type, ^a^*P* < 0.05; compared with CT type, ^b^*P* < 0.05.

**Table 5:** Relationship between SLC2A2 genotype and metformin efficacy (HbA1c value) in T2DM patients (*X* ± *S*).

Genotype	Number of cases	HbA1c		t value	*P* value
		Before treatment	After treatment		
TT	68	8.95 ± 1.56	8.07 ± 1.34	0.591	0.265
CT	30	8.91 ± 1.38	7.13 ± 1.15	5.125	0.000
CC	12	9.05 ± 1.31	5.15 ± 0.89	15.694	0.000
F value		1.236	48.695		
*P* value		0.346	0.000		

*Note.* FPG is fasting plasma glucose, 2hPBG is 2h postprandial blood glucose, HbA1c is hemoglobin A1c; compared with TT type, ^a^*P* < 0.05; compared with CT type, ^b^*P* < 0.05.

## Data Availability

The datasets used and analyzed during this study are available from the corresponding author upon reasonable request.
